RETRACTED

# Genetic association between asthma and alopecia areata: A two‐sample Mendelian randomization study

**DOI:** 10.1111/srt.13844

**Published:** 2024-07-04

**Authors:** Wenqian Du, Ke He, Xinyi Liu, Tingyi Yin, Shengxiang Xiao, Yan Zheng

**Affiliations:** ^1^ Department of Dermatology The First Affiliated Hospital of Xi'an Jiaotong University Xi'an China; ^2^ Department of Dermatology The Second Affiliated Hospital of Xi'an Jiaotong University Xi'an China

**Keywords:** alopecia areata, asthma, causal relationship, mendelian randomization

## Abstract

**Background:**

Many patients with asthma experience alopecia areata (AA) in their lives. However, it is unclear whether asthma causes or results from AA. Our objective was to investigate the genetic causal relationship between asthma and AA.

**Methods:**

Two‐sample Mendelian randomization (MR) was used to assess the causal relationship between asthma and AA based on the largest publicly available genome‐wide association study summary statistics. Androgenetic alopecia (AGA) and cicatricial alopecia (CA) were chosen as the control groups for AA. The main estimates were obtained using inverse variance weighting meta‐analysis (IVW), Mendelian randomization‐Egger (MR‐Egger), maximum likelihood estimation, and the weighted median. Sensitivity analyses were conducted using Cochran's Q test, MR‐Egger, and leave‐one‐out methods. Lastly, we conducted a reverse MR analysis to evaluate the possibility of reverse causation.

**Results:**

Genetically, asthma is associated with an increased risk of AA, while the association between genetically predicted AGA or CA and asthma was negative. The risk of AA increased by 1.86 times in patients with asthma under the IVW method (OR = 1.86, 95% CI = 1.31–2.629, *p* < 0.001). The reverse MR analysis did not find evidence supporting reverse causality from three phenotypes of alopecia to asthma. Sensitivity analyses yielded consistent causal estimates.

**Conclusion:**

This study suggests that asthma is causally associated with AA. The findings deepen our understanding of the role of asthma in the pathology of AA, which emphasizes the potential for opening a new vista for the prevention and diagnosis of AA.

## 1 INTRODUCTION

Alopecia areata (AA) is an autoimmune disease characterized by transient, non‐scarring hair loss and hair follicle preservation. Clinical severity ranges from small patches of hair loss to diffuse or total hair loss. AA affects almost 2% of the general population.^1^ The exact mechanisms of alopecia areata are still under investigation. Complex genetic susceptibility,^2^ oxidative stress injury,^3^ environmental factors,^4^ lifestyle,^5^ and advanced age contribute cooperatively to the occurrence and severity of AA,^6^ among which autoimmune and allergic diseases may play an important role in its pathological changes.^7^

RETRACTED

Asthma is one of the most common chronic non‐communicable diseases in the world, characterized by variable airflow limitation and respiratory symptoms.^8^ Autoimmunity and allergy play a major role in its development. Studies have reported an association between AA and asthma.^9^ Asthma was one of the most common comorbidities in patients with AA reported in a US retrospective cross‐sectional study.^10^ However, the relationship between asthma and AA has not been well studied. Therefore, we used Mendelian randomization (MR) to determine whether there is a causal relationship between asthma and AA.

MR is an instrumental variable (IV) analysis method that uses single nucleotide polymorphisms (SNPs) from genome‐wide association study (GWAS) as instruments, which are representative of the exposure characteristics, to detect causal relationships between complex characteristics, provided the necessary assumptions are met.^11^ IVs are not correlated with random error (the presence of variation such as age, sex, and weight, which must be adjusted for in observational studies) because SNP assignment follows the Mendelian inheritance rule, suggesting random assignment during the formation of a fertilized ovum.^12^ Therefore, the basic principle of MR research based on the SNP acting as an IV is comparable to that of randomized controlled trials. This strategy is relatively convenient, cost‐effective, and less likely to be confounded by covariates.^13^

In this study, we used available summary statistics from open‐access GWAS databases to perform a two‐sample MR analysis and evaluate the causality between asthma and AA. In order to investigate the relationship between asthma and alopecia areata in more detail and to further explore the mechanism of association between asthma and alopecia areata, we selected androgenetic alopecia (AGA) and cicatricial alopecia (CA) as control groups. The results of the current study may partly explain the underlying mechanism of AA and provide support for the future development of prevention and intervention strategies.

## 2 MATERIALS AND METHODS

### 2.1 Study design and data source

We performed a Mendelian randomization analysis to investigate the causal effects of asthma on AA and other types of alopecia. The IVs used for the MR study should meet the following three assumptions^11^:

1. The trait is strongly and robustly associated with the exposure of interest;
2. There are no confounders in the association between IVs and outcomes;
3. IVs do not affect the outcome except through their effect on the exposure (Figure 1).

RETRACTED

**FIGURE 1:** Assumptions and research design for Mendelian randomization analysis. (A) In order to verify the existence of causal correlation, it is necessary to meet the conditions as follows: (1) The trait is strongly and robustly associated with the exposure of interest; (2) There are no confounders of the association between IVs and outcome; (3) IVs does not affect the outcome except through its effect on the exposure. (B) Flowchart of Mendelian randomization analysis and sensitivity analyses. SNPs, single nucleotide polymorphisms; GWAS, genome‐wide association study; AA, Alopecia areata; AGA, Androgenic alopecia; CA, Cicatricial alopecia; IVs, instrumental variables; IVW, inverse variance weighting.

The MR approach uses genetic variants, which are randomly assigned at meiosis and therefore independent of potential confounders that bias observational studies, as proxies for a risk factor in an instrumental variable analysis. In our study, single nucleotide polymorphisms (SNPs) closely associated with traits were selected as IVs using summary data from open‐access GWAS from different independent studies with less sample overlap. Ethical approval was obtained for these studies. Summary statistics of GWAS for asthma were obtained from the open‐access GWAS website(https://gwas.mrcieu.ac.uk/) including 408442 European participants, while data for AA, AGA, and CA were obtained from the FinnGen biobank^14^ (https://www.finngen.fi/). The SNPs as IVs of exposure and outcome were all derived from GWAS of European ancestry to minimize potential bias from population heterogeneity. Details of the data sources are shown in Table 1.

**TABLE 1:** Data source and description.

ID	Trait	Population	Sample size	No. of cases	No. of control
ebi‐a‐GCST90014325	Asthma	European	408,442	56,167	352,255
finn‐b‐L12_ALOPECAREATA	Alopecia areata	European	211,139	289	210,850
finn‐b‐L12_ALOPECANDRO	Androgenic alopecia	European	119,087	98	118,989
finn‐b‐L12_HAIRLOSSSCAR	Cicatricial alopecia	European	211,139	80	211,059

To satisfy assumption 1, we selected SNPs strongly associated with asthma based on the genome‐wide significance threshold of *p* = 5e^−8^. Linkage disequilibrium clustering with a threshold of *r* ^2^ < 0.001 and a window size of 10,000 kb was used to determine whether the SNPs were genetically linked or not, with an *F*‐statistic > 10 used as a threshold for sufficient power, representing a 10% relative bias toward the null in the two‐sample MR setting.^15^ In this study, we also used the I^2^ statistic (the threshold was 90%) to assess the suitability of pooled data for two‐sample Mendelian randomization analyses.^16^ A higher I^2^ statistic means less bias due to weak instruments. We also removed SNPs associated with potential confounders of the outcome of interest according to the PhenoScanner V2 database.^17^

RETRACTED

### 2.2 Statistical analyses

Main estimates were obtained using inverse variance weighting (IVW), weighted median, Mendelian randomization Egger (MR‐Egger)^18^ ^,^ and Maximum Likelihood.^19^ Random‐effects IVW was used when there was heterogeneity between the SNPs included in each analysis. Otherwise, a fixed effects IVW model was used. This method provided the highest statistical power and also accounted for balanced pleiotropy when the above MR assumptions were met. The weighted median used most SNPs (majority of genetic variants) to determine the presence or absence of causality. MR‐Egger regression was mainly used to assess horizontal pleiotropy and provide the *I* ^2^ statistic to assess weak instrumental variable bias. Maximum likelihood was used to assess bias due to sample overlap.^20^

Sensitivity analyses were performed to assess heterogeneity, pleiotropy, and outlier SNPs.^21^ The Cochran *Q* statistic was used to test for heterogeneity. A *p* value < 0.05 was considered to indicate statistically significant heterogeneity. The presence of horizontal and directional pleiotropy violated assumption 3. The intercept in the MR‐Egger analysis was used to assess directional pleiotropy. If the intercept was not significantly different from zero (*p* > 0.05), the pleiotropy effect could be ignored.^18^ The leave‐one‐out test was used to assess the influence of outliers. Scatterplots, forest plots, and funnel plots were created to further demonstrate the sensitivity of the results. Finally, a reverse MR analysis was performed to evaluate the possibility of reverse causation.

All statistical analyses were performed using the “two‐sample MR” and “Mendelian randomization” packages in R software (version 4.3.2).

## 3 RESULTS

### 3.1 Genetically asthma is associated with increased risk of AA, but not with AGA and CA

During instrumental variable clumping, no SNPs were associated with confounding factors and outcomes, 1 SNP (rs35320232) was removed for incompatible alleles and 1 SNP (rs13099273) was removed for being palindromic with intermediate allele frequencies. Finally, 78 asthma‐related SNPs that met the three main assumptions of the MR study were retained for further analysis (Table S1). The *F*‐statistic value of all SNPs was above 10. *I* ^2^ statistic was 90.4% which meant low weak instruments bias in further analysis.

We used the two‐sample MR method to evaluate the potential causal relationship between asthma and AA. The MR analyses suggested a causal relationship between asthma and AA. The risk of AA increased in patients with asthma under the fixed effects IVW method (OR = 1.859, 95% CI = 1.315−2.629, *p* < 0.001). The causal association was confirmed using both maximum likelihood estimation (OR = 1.817, 95% CI = 1.288−2.565, *p* = 0.001) and the weighted median method (OR = 2.365, 95% CI = 1.383−4.045, *p* = 0.002) (Figure 2). When we set the rate of sample overlap as 60%, the causal relationship still existed (OR_psi0.6_ = 1.212, 95% CI _psi0.6_ = 1.036−2.195, p _psi0.6_ = 0.033).

RETRACTED

**FIGURE 2:** Main estimates of Mendelian randomization between asthma and types of alopecia. nSNP, number of single nucleotide polymorphisms; OR, odds ratio; CI, confidence interval; AA, alopecia areata; AGA, androgenic alopecia; CA, cicatricial alopecia; IVs, instrumental variables; IVW, inverse variance weighting; ML, maximum likelihood; WM, weighted median.

However, we assessed the relationship between asthma and AGA, as well as asthma and CA, using the same MR methods. The results of the fixed effects IVW, the MR‐Egger, the weighted median, and the maximum likelihood estimation suggested that there was no clear causal relationship between genetically predicted asthma and the risk of AGA and CA, with all *p* values greater than 0.05 (Figure 2).

The scatter plots demonstrate the impact of the 76 SNPs on asthma and AA, as well as on AGA and CA (Figure 3A–C). The funnel plots illustrate the distribution of the effect of a single SNP (Figure S1A–C), while the forest plots display the effect of an individual SNP on the estimation of the outcomes (Figure S1D–F).

**FIGURE 3:** Scatter plots about the causal effect of asthma on types of alopecia. (A) Scatter plots about the causal effect of asthma on alopecia areata. (B) Scatter plots about the causal effect of asthma on androgenic alopecia. (C) Scatter plots about the causal effect of asthma on cicatricial alopecia.

### 3.2 Sensitivity analysis

The analysis did not reveal any significant heterogeneity among the asthma‐related SNPs (Cochran's *Q* statistic was 80.441, *p* = 0.285, MR‐Egger method). Furthermore, the MR‐Egger intercept analysis found no evidence of directional pleiotropy (egger intercept = −0.019, *p* = 0.537) in MR analysis between asthma and AA, suggesting that potential confounding factors through other pathways were unlikely to affect the exposure‐outcome relationship (Table 2).

**TABLE 2:** Sensitive analysis for heterogeneity, pleiotropy and outlier SNPs.

Exposure	Outcome	Heterogeneity			Pleiotropy			The leave‐one‐out test
		method	*Q*	*Q*_*p* value	Egger_intercept	Standard error	*p* value	outliers
Asthma	AA	MR Egger	80.441	0.285	‐0.019	0.030	0.537	NA
		IVW	80.858	0.301				
Asthma	AGA	MR Egger	76.543	0.397	0.013	0.051	0.795	NA
		IVW	76.614	0.427				
Asthma	CA	MR Egger	76.777	0.390	0.033	0.056	0.559	NA
		IVW	77.135	0.410				
AA	Asthma	MR Egger	26.139	0.002	0.003	0.008	0.748	NA
		IVW	26.457	0.003				
AGA	Asthma	MR Egger	0.683	0.711	0.009	0.007	0.362	NA
		IVW	2.055	0.561				
CA	Asthma	MR Egger	3.988	0.781	0.002	0.004	0.717	NA
		IVW	4.130	0.845				

Abbreviations: AA, alopecia areata; CA, cicatricial alopecia; AGA, androgenic alopecia; IVW, inverse variance weighting.

RETRACTED

The leave‐one‐out analysis indicated that no single SNP had a significant effect on the results, suggesting the robustness and reliability of the MR studies (Figure S1G–I). The reverse MR analysis did not find any evidence supporting reverse causality from three phenotypes of alopecia to asthma (Table S2, Figures S2 and S3).

## 4 DISCUSSION

Alopecia, or hair loss, is a disease that affects a significant number of people worldwide and is associated with psychological disorders.^22^ There are two main types of alopecia: CA and non‐cicatricial alopecia. The most common types of non‐cicatricial alopecia are AA and AGA. The causes of alopecia are complex and involve multiple factors. Autoimmune and inflammatory diseases, including asthma, may contribute to alopecia. To our knowledge, this is the first MR study to investigate the potential causal relationship between asthma and alopecia. Our study showed that genetically predicted asthma increases the risk of AA later in life, but not of AGA and CA. The results were supported by consistent magnitude and direction of robust methods.

AGA, also known as male‐pattern alopecia, is the most common type of alopecia.^23^ It is characterized by progressive terminal hair loss after puberty, and its incidence and prevalence depend on race and age. At least 80% of men and 50% of women are affected by the age of 70 years. The progression of AGA is mainly contributed by genetics and sensitivity to androgens,^24^ with testosterone being a major androgen that is converted to dihydrotestosterone (DHT) by 5α‐reductase. DHT binds to androgen receptors in hair follicles, causing them to shrink and shortening their anagen cycle, ultimately resulting in hair loss.^25^ Some metabolic disorders may also have an influence on AGA by elevating androgens or other metabolites.^26^ It is important to note that the pathogenesis of AGA differs from that of AA, which is primarily considered an autoimmune disease. This may explain why no association was found between asthma and AGA.

Scarring alopecia, also known as CA, is divided into primary and secondary forms. It is characterized by irreversible inflammation and damage to the hair follicles, resulting in scarring and hair loss. Primary CA is primarily caused by direct inflammatory attacks on hair follicles by various inflammatory infiltrates, such as lymphocytes, neutrophils, and mixed cells. This can occur in diseases such as chronic cutaneous lupus erythematosus, lichen planopilaris, folliculitis decalvans, and folliculitis (acne) necrotica.^27^ Secondary CA results from the random destruction of hair follicles due to inflammatory processes or mechanical damage, such as trauma, burns, radiation, infections, or tumors.^28^ While autoimmune and inflammatory diseases can cause CA, the pathogenesis of CA differs from that of non‐cicatricial alopecia. Our results demonstrate that asthma does not increase the risk of CA, indicating that asthma may not cause CA.

RETRACTED

Previous observational studies have shown that AA is associated with autoimmune and inflammatory diseases, including asthma. A Danish nationwide register‐based cohort study found that asthma occurred more frequently in patients with AA compared to controls.^9^ Similarly, a population‐based study including 51,561 cases with AA and 51,410 matched controls found that the prevalence of asthma was significantly higher in patients with AA than in the control group.^29^ Furthermore, a recent retrospective cohort study based on US claims data demonstrated that the incidence of asthma was higher in individuals with African ancestry compared to those without (12.8% vs. 8.8%, respectively).^7^ Although observational studies may be subject to recall bias, our study was based on a large GWAS dataset and a restricted population to minimize bias. Our findings are consistent with previous research, indicating that asthma is a risk factor for African ancestry. No observational studies have shown an association between asthma and AGA or CA.

The association between asthma and AA is not well understood, but there are some mechanisms that can explain the connection. An explanation is the presence of genetic variants in immune‐related genes that have been linked to both conditions. Previous studies have shown that the cytotoxic T‐lymphocyte protein 4 (CTLA‐4) gene polymorphism is associated with asthma.^30^, ^31^ CTLA‐4 is expressed on activated T cells and is involved in T cell activation and differentiation, which plays an important role in autoimmune diseases. Studies have also demonstrated a genetic variant association of CTLA‐4 with AA.^32^ Other genetic variants, such as HLA‐DRB1 and PTPN22, are associated with an increased susceptibility to asthma and AA.^33^ This supports the association between asthma and AA in the present study. Additionally, both asthma and AA are considered autoimmune diseases, suggesting that they may share similar pathogenesis and immune pathways. Th2 cells play an essential role in the pathogenesis of asthma. They produce IL‐4, IL‐5, and IL‐13 under adaptive immune response, leading to airway obstruction and hyperresponsiveness.^34^ These cytokines are also involved in AA pathogenesis, as levels of IL‐4, IL‐5, and IL‐13 have been found to be elevated in the lesions or serum/blood of patients with AA.^35^ Several clinical trials have shown that Dupilumab, a monoclonal antibody that targets IL‐4 and IL‐13, is effective in treating asthma.^36^, ^37^ Recent studies have also demonstrated its effectiveness in treating AA and indicated the involvement of the Th2 pathway in AA pathogenesis.^38^, ^39^ In addition, Th1 and Th17 cells also play an important role in asthma, particularly in those with lower Th2 immune response, mainly producing IFN‐γ, IL‐17, and IL‐22. Patients with AA also exhibit elevated levels of Th1 and Th17‐related cytokines, which are essentially involved in the pathogenesis of AA.^40^, ^41^ The changes in immune system may cause a breakdown of immune privilege of hair follicles, which have been thought to be a crucial driver of AA.^1^, ^42^ These mechanisms may form the foundation of causal association between asthma and AA.

RETRACTED

Our study has several strengths. First, the MR concept is less susceptible to unobserved confounding and reverse causality, which are issues in observational studies. Second, we conducted outlier assessment and a wide range of sensitivity analyses that accounted for different patterns of pleiotropy, which increased the robustness of the results and strengthened the evidence of our findings. There are still shortcomings in our research. First, MR studies have some disadvantages compared to randomized clinical trials, such as lack of stability of subjects or weak controllability of studies. Second, the number of cases from summary data used in this study was lower than anticipation, which is attributed to low incidence of alopecia areata. Additionally, due to the lack of suitable summary‐level data, sex‐specific and ethnic‐stratified analyses were not possible. Future high‐quality randomized controlled studies based on large sample sizes are still needed to further verify this association.

## 5 CONCLUSION

This study suggests that asthma has a positive effect on AA, while it has no association with the risk of AGA and CA. Furtherly exploration into the role of asthma in AA will promote an understanding of its pathogenesis. The findings enhance our comprehension of the relationship between asthma and the pathology of AA, highlighting the possibility of new avenues for the prevention and diagnosis of AA.

RETRACTED

## CONFLICT OF INTEREST STATEMENT

The authors declare that the research was conducted in the absence of any commercial or financial relationships that could be construed as a potential conflict of interest.

## Supporting information

Supplementary Material

## Data Availability

The study's original contributions are partially included in the article and Supplementary Materials. For further inquiries, please contact the corresponding author.

## References

[1] Pratt CH , King LE , Messenger AG , Christiano AM , Sundberg JP . Alopecia areata. Nat Rev Dis Primer. 2017;3:17011. doi:10.1038/nrdp.2017.11 PMC557312528300084

[2] Oka A , Takagi A , Komiyama E , et al. Alopecia areata susceptibility variant in MHC region impacts expressions of genes contributing to hair keratinization and is involved in hair loss. EBioMedicine. 2020;57:102810. doi:10.1016/j.ebiom.2020.102810 32580135 PMC7317227

[3] Peterle L , Sanfilippo S , Borgia F , Cicero N , Gangemi S . Alopecia areata: a review of the role of oxidative stress, possible biomarkers, and potential novel therapeutic approaches. Antioxidants. 2023;12(1):135. doi:10.3390/antiox12010135 36670997 PMC9854963

[4] Touil H , Mounts K , De Jager PL . Differential impact of environmental factors on systemic and localized autoimmunity. Front Immunol. 2023;14:1147447. doi:10.3389/fimmu.2023.1147447 37283765 PMC10239830

[5] Minokawa Y , Sawada Y , Nakamura M . Lifestyle factors involved in the pathogenesis of alopecia areata. Int J Mol Sci. 2022;23(3):1038. doi:10.3390/ijms23031038 35162962 PMC8835065

[6] Simakou T , Butcher JP , Reid S , Henriquez FL . Alopecia areata: a multifactorial autoimmune condition. J Autoimmun. 2019;98:74‐85. doi:10.1016/j.jaut.2018.12.001 30558963

[7] George P , Jagun O , Liu Q , et al. Prevalence of autoimmune and inflammatory diseases and mental health conditions among an alopecia areata cohort from a US administrative claims database. J Dermatol. 2023;50(9):1121‐1128. doi:10.1111/1346-8138.16839 37291688

[8] Papi A , Brightling C , Pedersen SE , Reddel HK . Asthma. Lancet. 2018;391(10122):783‐800. doi:10.1016/S0140-6736(17)33311-1 29273246

[9] Egeberg A , Anderson S , Edson‐Heredia E , Burge R . Comorbidities of alopecia areata: a population‐based cohort study. Clin Exp Dermatol. 2021;46(4):651‐656. doi:10.1111/ced.14507 33175413

[10] Huang KP , Mullangi S , Guo Y , Qureshi AA . Autoimmune, atopic, and mental health comorbid conditions associated with alopecia areata in the United States. JAMA Dermatol. 2013;149(7):789‐794. doi:10.1001/jamadermatol.2013.3049 23700152

[11] Birney E . Mendelian randomization. Cold Spring Harb Perspect Med. 2022;12(4):a041302. doi:10.1101/cshperspect.a041302 34872952 PMC9121891

RETRACTED

[12] Sekula P , Del Greco M F , Pattaro C , Köttgen A . Mendelian randomization as an approach to assess causality using observational data. J Am Soc Nephrol JASN. 2016;27(11):3253‐3265. doi:10.1681/ASN.2016010098 27486138 PMC5084898

[13] Skrivankova VW , Richmond RC , Woolf BAR , et al. Strengthening the reporting of observational studies in epidemiology using Mendelian randomization: the STROBE‐MR statement. JAMA. 2021;326(16):1614‐1621. doi:10.1001/jama.2021.18236 34698778

[14] Kurki MI , Karjalainen J , Palta P , et al. FinnGen provides genetic insights from a well‐phenotyped isolated population. Nature. 2023;613(7944):508‐518. doi:10.1038/s41586-022-05473-8 36653562 PMC9849126

[15] Burgess S , Thompson SG , CRP CHD Genetics Collaboration . Avoiding bias from weak instruments in Mendelian randomization studies. Int J Epidemiol. 2011;40(3):755‐764. doi:10.1093/ije/dyr036 21414999

[16] Bowden J , Del Greco M F , Minelli C , Davey Smith G , Sheehan NA , Thompson JR . Assessing the suitability of summary data for two‐sample Mendelian randomization analyses using MR‐Egger regression: the role of the I2 statistic. Int J Epidemiol. 2016;45(6):1961‐1974. doi:10.1093/ije/dyw220 27616674 PMC5446088

[17] Kamat MA , Blackshaw JA , Young R , et al. PhenoScanner V2: an expanded tool for searching human genotype‐phenotype associations. Bioinformatics. 2019;35(22):4851‐4853. doi:10.1093/bioinformatics/btz469 31233103 PMC6853652

[18] Burgess S , Thompson SG . Interpreting findings from Mendelian randomization using the MR‐Egger method. Eur J Epidemiol. 2017;32(5):377‐389. doi:10.1007/s10654-017-0255-x 28527048 PMC5506233

[19] Yavorska OO , Burgess S . Mendelian randomization: an R package for performing Mendelian randomization analyses using summarized data. Int J Epidemiol. 2017;46(6):1734‐1739. doi:10.1093/ije/dyx034 28398548 PMC5510723

[20] Xue H , Shen X , Pan W . Constrained maximum likelihood‐based Mendelian randomization robust to both correlated and uncorrelated pleiotropic effects. Am J Hum Genet. 2021;108(7):1251‐1269. doi:10.1016/j.ajhg.2021.05.014 34214446 PMC8322939

[21] Burgess S , Bowden J , Fall T , Ingelsson E , Thompson SG . Sensitivity analyses for robust causal inference from Mendelian randomization analyses with multiple genetic Variants. Epidemiol Camb Mass. 2017;28(1):30‐42. doi:10.1097/EDE.0000000000000559 PMC513338127749700

[22] Workman K , Piliang M . Approach to the patient with hair loss. J Am Acad Dermatol. 2023;89(2S):S3‐S8. doi:10.1016/j.jaad.2023.05.040 37591563

[23] Ntshingila S , Oputu O , Arowolo AT , Khumalo NP . Androgenetic alopecia: an update. JAAD Int. 2023;13:150‐158. doi:10.1016/j.jdin.2023.07.005 37823040 PMC10562178

RETRACTED

[24] Saceda‐Corralo D , Domínguez‐Santas M , Vañó‐Galván S , Grimalt R . What's new in therapy for male androgenetic alopecia? Am J Clin Dermatol. 2023;24(1):15‐24. doi:10.1007/s40257-022-00730-y 36169916

[25] Devjani S , Ezemma O , Kelley KJ , Stratton E , Senna M . Androgenetic alopecia: therapy update. Drugs. 2023;83(8):701‐715. doi:10.1007/s40265-023-01880-x 37166619 PMC10173235

[26] Du Y , Lu C , Bi L , et al. Causal effects of genetically determined metabolites on androgenetic alopecia: a two‐sample Mendelian randomization analysis. Skin Res Technol. 2024;30(5):e13732. doi:10.1111/srt.13732 38747971 PMC11095465

[27] Bolduc C , Sperling LC , Shapiro J . Primary cicatricial alopecia: lymphocytic primary cicatricial alopecias, including chronic cutaneous lupus erythematosus, lichen planopilaris, frontal fibrosing alopecia, and Graham‐Little syndrome. J Am Acad Dermatol. 2016;75(6):1081‐1099. doi:10.1016/j.jaad.2014.09.058 27846944

[28] Kanti V , Röwert‐Huber J , Vogt A , Blume‐Peytavi U . Cicatricial alopecia. J Dtsch Dermatol Ges J Ger Soc Dermatol JDDG. 2018;16(4):435‐461. doi:10.1111/ddg.13498 29645394

[29] Kridin K , Renert‐Yuval Y , Guttman‐Yassky E , Cohen AD . Alopecia areata is associated with atopic diathesis: results from a population‐based study of 51,561 patients. J Allergy Clin Immunol Pract. 2020;8(4):1323‐1328.e1. doi:10.1016/j.jaip.2020.01.052 32036002

[30] Munthe‐Kaas MC , Carlsen KH , Helms PJ , et al. CTLA‐4 polymorphisms in allergy and asthma and the TH1/TH2 paradigm. J Allergy Clin Immunol. 2004;114(2):280‐287. doi:10.1016/j.jaci.2004.03.050 15316504

[31] Andiappan AK , Puan KJ , Sio YY , et al. Functional CTLA‐4 variants associate to both allergic asthma and rhinitis potentially by modulating naïve regulatory T cells. Allergy. 2022;77(9):2856‐2858. doi:10.1111/all.15386 35607825

[32] John KKG , Brockschmidt FF , Redler S , et al. Genetic variants in CTLA4 are strongly associated with alopecia areata. J Invest Dermatol. 2011;131(5):1169‐1172. doi:10.1038/jid.2010.427 21346773

[33] Moravvej H , Tabatabaei‐Panah PS , Abgoon R , et al. Genetic variant association of PTPN22, CTLA4, IL2RA, as well as HLA frequencies in susceptibility to alopecia areata. Immunol Invest. 2018;47(7):666‐679. doi:10.1080/08820139.2018.1480032 29979892

[34] Ji T , Li H . T‐helper cells and their cytokines in pathogenesis and treatment of asthma. Front Immunol. 2023;14:1149203. doi:10.3389/fimmu.2023.1149203 37377958 PMC10291091

[35] Passeron T , King B , Seneschal J , et al. Inhibition of T‐cell activity in alopecia areata: recent developments and new directions. Front Immunol. 2023;14:1243556. doi:10.3389/fimmu.2023.1243556 38022501 PMC10657858

RETRACTED

[36] Castro M , Corren J , Pavord ID , et al. Dupilumab efficacy and safety in moderate‐to‐severe uncontrolled asthma. N Engl J Med. 2018;378(26):2486‐2496. doi:10.1056/NEJMoa1804092 29782217

[37] Bacharier LB , Maspero JF , Katelaris CH , et al. Dupilumab in children with uncontrolled moderate‐to‐severe asthma. N Engl J Med. 2021;385(24):2230‐2240. doi:10.1056/NEJMoa2106567 34879449

[38] Guttman‐Yassky E , Renert‐Yuval Y , Bares J , et al. Phase 2a randomized clinical trial of dupilumab (anti‐IL‐4Rα) for alopecia areata patients. Allergy. 2022;77(3):897‐906. doi:10.1111/all.15071 34460948 PMC9997752

[39] Renert‐Yuval Y , Pavel AB , Del Duca E , et al. Scalp biomarkers during dupilumab treatment support Th2 pathway pathogenicity in alopecia areata. Allergy. 2023;78(4):1047‐1059. doi:10.1111/all.15561 36271804 PMC11344221

[40] Loh SH , Moon HN , Lew BL , Sim WY . Role of T helper 17 cells and T regulatory cells in alopecia areata: comparison of lesion and serum cytokine between controls and patients. J Eur Acad Dermatol Venereol JEADV. 2018;32(6):1028‐1033. doi:10.1111/jdv.14775 29283462

[41] Waśkiel‐Burnat A , Osińska M , Salińska A , et al. The role of serum Th1, Th2, and Th17 cytokines in patients with alopecia areata: clinical implications. Cells. 2021;10(12):3397. doi:10.3390/cells10123397 34943905 PMC8699846

[42] Xu W , Shen Y , Sun J , Wei D , Xie B , Song X . Causal role of immune cells in alopecia areata: a two‐sample Mendelian randomization study. Skin Res Technol. 2024;30(1):e13579. doi:10.1111/srt.13579 38221794 PMC10788640

